# High-Throughput Sequencing Investigation of Bacterial Diversity in Chronic Suppurative Otitis Media and Middle Ear Cholesteatoma

**DOI:** 10.1155/2022/9616582

**Published:** 2022-09-19

**Authors:** Xiuqin Cheng, Abulajiang Tuoheti, Xiaobang Huang, Xingzhi Gu

**Affiliations:** ^1^Diagnosis and Treatment Center of Otorhinolaryngology, People's Hospital of Xinjiang Uygur Autonomous Region, Urumqi, Xinjiang Uygur Autonomous Region, China; ^2^Department of Otorhinolaryngology Head and Neck Surgery, Tianjin Beichen Hospital, Tianjin, China; ^3^Otorhinolaryngology & Head and Neck Surgery, Sanya Central Hospital (Hainan Third People's Hospital), Sanya, Hainan, China

## Abstract

**Background:**

Chronic otitis media is a common middle ear disease in otolaryngology. Bacterial infection is considered as the cause of the disease, but relying on conventional bacterial cultures can be problematic for identifying specific pathogens. Current research suggests that bacteria in microbial communities can only be identified by rDNA sequencing of bacteria.

**Methods:**

This cross-sectional study utilized broad-range PCR amplification of 16S rRNA genes with clone analysis to compare bacterial diversity in lesions from 6 patients with chronic suppurative otitis media (CSOM) and 10 patients with cholesteatoma of middle ear lesions. Bacteria were analyzed at the levels of phylum, order, family, genus, and species.

**Results:**

The age and sex difference between the patients with chronic suppurative otitis media and the patients with middle ear cholesteatoma were comparable (*P* > 0.05). Bacterial species abundance and species diversity were greater in cholesteatoma of the middle ear lesions than in CSOM lesions. The total number of detected operational taxonomic units (OTU) was 838, comprising 788 OTU detected in cholesteatoma pathological tissues, 230 in CSOM pathological tissues, and 180 OTU common to both groups. Proteus is a major part of CSOM (99.46%, *P* = 0.000321). The phyla detected in the Cholesteatoma samples were Proteus (Proteobacteria) (35.77%), thikum (Firmicutes) (44.21%, *P* = 0.001071), and Actinomycetes (Actinobacteria) (16.66%, *P* = 0.032464). At all bacterial taxonomic levels, the epithelial tissue of middle ear cholesteatoma was complex in terms of bacterial diversity, covering many Gram-positive and Gram-negative bacteria, likely related to bacterial microbiome formation. In contrast, the bacteriology of the CSOM lesions was relatively simple at all taxonomic levels, with all sequences characterized as belonging to Gram-negative bacteria.

**Conclusion:**

Our results suggest that persistent middle ear cholesteatoma infection may be a microbial flora disorder related to conditional pathogenic bacteria rather than a single bacterial infectious disease. The pathogen is relatively single in the diseased tissue of chronic suppurative otitis media, which is the main reason for its effective antiinfection treatment.

## 1. Introduction

Chronic otitis media, a common disease in otorhinolaryngology, is caused by inflammatory lesions in the middle ear and mastoid cavity and is characterized by ear discharge (otorrhea) and hearing loss. Some patients experience life-threatening complications [1, 2]. Clinically, chronic otitis media refers to chronic suppurative otitis media (CSOM) and middle ear cholesteatoma. Bacterial infection is the main pathogenic factor in chronic otitis media [3].

Bacterial culture of the external ear canal secretions is often used to confirm the presence of pathogenic bacteria, and various pathogenic bacteria, including methicillin-resistant *Staphylococcus aureus*, have been obtained through this method [4].

Although sensitive antimicrobial agents based on culture results have been successfully used to treat patients, some cases of ineffective treatments have still been reported [5, 6]. Studies have confirmed that bacterial biofilm formation leading to resistance to antimicrobial agents may be among the reasons for the persistent symptoms in some patients [7–10]. Bacterial culture results are affected by many factors, including the inability of some bacteria to grow on standard medium and restrictions on specimen collection. Thus, in some cases, it is not easy to identify and treat the causative pathogen [11] successfully.

In recent years, there have been numerous reports on molecular techniques for the study of bacteria of otitis media. Previous work did not report any bacteria isolated from the middle ear secretions of children and adults by conventional bacterial culture methods. However, it confirmed that gene sequencing resulted in the isolation of various bacterial sequences, including the phylum and the genus Grapevine [12]. Neeff et al. demonstrated that analysis of CSOM and healthy human middle ear mucosa through molecular techniques could be accurately used to assess microbial communities in the middle ear or mastoid mucosa [13]. However, there are limited reports on the distribution of microbes in different types of chronic otitis media.

The current study used 16S rRNA gene amplicon sequencing to study microbial communities in CSOM and cholesteatoma of middle ear (CME) diseased tissues. Differences in microbial species abundance, diversity, and levels of phylum, class, order, family, genus, and species were compared. These analyses provide a basis for future studies on the characterization of bacteria at the molecular level in chronic otitis media.

## 2. Materials and Methods

### 2.1. Patient Information

All patients in this study had chronic otitis media and received surgical treatment in the otolaryngology department of Xinjiang Uygur Autonomous Region People's Hospital from January 2017 to June 2019. Among the 16 eligible patients, six cases were chronic suppurative otitis media, and 10 were middle ear cholesteatoma. None of the patients used antibiotic ear drops or systemic antibiotics before surgery, but according to the requirement for preventive use of antibiotics, all patients received intravenous cephalosporins 30 min∼2 h before surgery. Patients were not associated with basic metabolic diseases such as diabetes or rheumatism and did not have external auditory canal fungal infections. The age and sex between the patients with chronic suppurative otitis media and the patients with middle ear cholesteatoma were comparable (*P* > 0.05).

The study was approved by the Ethics Committee of the People's Hospital of the Xinjiang Uygur Autonomous Region (Xinjiang District Hospital Ethics Committee 2015054). The patients or their authorized families had signed the informed consent.

The operation mode of canal wall up [CWU] tympanic forming or canal wall down [CWD] tympanic forming was selected according to the disease severity of the patient. After opening the tympanic sinus and mastoid cavity during the operation, the middle ear lesion tissue was retained (after cleaning the matrix, the epithelium and granulation tissue of cholesteatoma were retained). Following the collection of pathological tissues, the accompanying blood and floats were washed with normal saline, immediately placed into a specimen tube, frozen in liquid nitrogen, and then stored at −80°.

### 2.2. Absolute Quantification of 16S rRNA Amplicon Sequencing

Absolute quantification of 16S rRNA amplicon sequencing was performed by Genesky Biotechnologies Inc. (Shanghai, 201315, China). Briefly, total genomic DNA was extracted using a Fast DNA SPIN Kit for Soil (MP Biommedicals, Santa Ana, CA, USA) according to the manufacturer's instructions. The integrity of the genomic DNA was assessed through agarose gel electrophoresis, and the concentration and purity of genomic DNA were measured using a NanoDrop 2000 spectrophotometer and a Qubit 3.0 fluorometer.

The GC content was artificially synthesized. An appropriate proportion of spike-in mixture with known gradient copy numbers was then added to the sample DNA. The V3-V4 hypervariable regions of the 16s rRNA gene and spike-ins were amplified with the primers xxxF (5′-CCTACGGGNGGCWGCAG-3′) and xxxR (5′-GACTAACHVGGGTATCTAATCC-3′) and then sequenced using an Illumina NovaSeq 6000 sequencer.

### 2.3. Sequence Data Processing and Analysis

Raw read sequences were processed in QIME2 [14]. The adaptor and primer sequences were trimmed using the cutadapt plugin, and the DADA2 plugin was used for quality control and to identify amplicon sequence variants (ASVs) [15]. Taxonomic assignments of representative ASVs were performed with a confidence threshold of 0.8 by a pretrained Naive Bayes classifier trained on the Greengenes database (version 13.8). The spike-in sequences were then identified, and reads were counted. A standard curve for each sample was generated based on the read counts versus spike-in copy number, and the absolute copy number of ASVs in each sample was calculated using the read counts of the corresponding ASV. Since the spike-in sequence is not a component of the sample flora, the spike-in sequence was removed in the subsequent analysis [16].

## 3. Results

### 3.1. Analysis of Species Abundance and Diversity

High-throughput 16SrRNA gene sequencing technology was used to sequence samples from 16 patients with CSOM or cholesteatoma. A total of 4,672,171 raw sequences reads and 3,415,184 optimized sequence reads were obtained from the 16 patients with middle ear lesions (6 CSOM cases and 10 cholesteatoma cases). The average sequence length from the total of 1,243,460,816 bases was 364.10 bp.

The sequences obtained from each patient group were 582,102 and 1,485,436 for CSOM and cholesteatoma, respectively.

### 3.2. Taxonomic Analysis of Pathological Tissue Flora from Patients with CSOM or Cholesteatoma

A total of 833 operational taxonomic units (OTU) were subjected to taxonomic classification, and 28 phyla, 50 classes, 63 orders, 128 families, 264 genera, and 232 species were identified and further analyzed.

Samples from different disease groups have certain common characteristics. Based on the OTU abundance table, each group's unique OTU and common OTU were screened and visualized. The total number of detected OTU was 838, comprising 788 OTU detected in cholesteatoma pathological tissues, 230 in CSOM pathological tissues, and 180 OTU common to both groups (Figure 1).

### 3.3. Phylum

Bacterial community analysis at the phylum level revealed that the community flora of CSOM tissues was simpler than that of Cholesteatoma samples. The phylum *Proteus (Proteobacteria)* was detected in both groups. The results confirmed that Proteus is a major part of CSOM (99.46%, *P*=0.000321). In addition, the proteus phylum members such as *Pseudomonas aeruginosa* and *Escherichia coli* are the common Gram-negative pathogens. The microbial community of Cholesteatoma samples was more complex. The phyla detected in the Cholesteatoma samples were Proteus (*Proteobacteria*) (35.77%), thikum (*Firmicutes*) (44.21%, *P*=0.001071), and *Actinomycetes* (*Actinobacteria*) (16.66%, *P*=0.032464). Thikum and Actinomycetes formed most Gram-positive bacteria (Figure 2).

### 3.4. Class

Bacterial sequence analysis at the class level showed statistically significant differences between the two groups (CSOM and cholesteatoma) in the classes *Gammaproteobacteria γ*-Proteus (*P*=0.03), *Bacilli* (*P*=0.01034), *Clostridia* (*P*=0.034), and *Bacteroidia* (*P*=0.041). In general, the measured species of the cholesteatoma lesions were higher than those of the CSOM group, indicating that the abundance of microbes was greater. In the CSOM group, *Gammaproteobacteria γ*- and *β*- Proteus (*Betaproteobacteria*) were predominantly detected, indicating that the number of microbial species present at the class level is relatively small in this group (Figure 3).

### 3.5. Order

At the order level, *Pseudomonadales* and *Burkholderiales* have an absolute advantage in CSOM, with *Pseudomonadales* being statistically significant (*P*=0.00129). *Pseudomonas aeruginosa* strain PAO was identified in the bacterial species map at the sample sequencing level. In the cholesteatoma group, the statistically significant orders were *Bacillales* (*P*=0.011887), *Clostridiales* (*P*=0.011887), and *Bacteroidales* (*P*=0.002532). The description of the bacterial communities at the order level also suggests that cholesteatoma is more complex in bacterial diversity (Figure 4).

### 3.6. Family

Analysis of sequencing results at the family level indicated that *Pseudomonadaceae* (37.74%), *Moraxellaceae* (35.13%), and *Alcaligenaceae* (26.13%) were predominant in the CSOM samples. In particular, the detection of *Pseudomonadaceae* (*P*=0.000976) was statistically significant. Bacterial diversity at the family level in the cholesteatoma group was more complex than that of the CSOM group. Families with broad coverage in the cholesteatoma group were *Staphylococcaceae* (33.53%), *Enterobacteriaceae* (22.93%), *Brevibacteriaceae* (8.49%), *Pseudomonadaceae* (8.39%), and *Corynebacteriaceae* (6.31%). The statistically significant families *Porphyromonadaceae* and *Lachnospiraceae* are mostly conditional pathogenic bacteria (Figure 5).

### 3.7. Genus

Sequencing analysis of bacterial communities of CSOM and cholesteatoma lesions at the genus level revealed that 16 genera, including “Others” and “No_Rank,” were detected across the two groups. However, only *Pseudomonas* was detected in both groups and showed a statistically significant difference in relative abundance between the two groups (*P* = 0.000601). *Pseudomonas* was significantly higher in the CSOM (37.74%) than in the middle ear cholesteatoma group (8.39%). Other genera detected in the CSOM group were *Acinetobacter* (35.13%) and *Alkaligenes* (26.02%) (Figure 6). Gram-negative genera were dominant. These genera include *Pseudomonas aeruginosa*, *Acinetobacter baumannii*, and fecal alkaloid bacteria, which are the most common resistant strains of nosocomial infections. In contrast, the composition of bacterial genera of the cholesteatoma group was more elaborate, comprising *Staphylococcus* (33.53%), *Providencia* (12.34%), Others (9.56%), *Proteus* (9.05%), *Brevibacterium* (8.49%), *Pseudomonas* (8.39%), *Corynebacterium* (6.31%), *Finegoldia* (2.74%), No_Rank (2.15%), *Achromobacter* (2.09%), *Clostridium* (1.53%), *Tissierella* (1.32%), *Enterococcus* (1.26%), and *Ralstonia* (1.08%) (Figure 6). These genera are diverse and include Gram-positive and Gram-negative bacteria, cocci, bacilli, and aerobic and anaerobic bacteria.

### 3.8. Species

Sequencing analysis at the species level demonstrated that the pathogenic bacterial species composition in cholesteatoma lesions was more complex than in the CSOM lesions, while many more types of pathogenic bacteria were detected in the cholesteatoma group than in the CSOM group. The statistical results of the uncultured organism was *P*=0.001476 while and the uncultured-bacterium was *P*=0.0043290. The detection rate of *Pseudomonas aeruginosa* in the CSOM group was much higher than that in the middle ear cholesteatoma group (*P*=0.000576, Figure 7).

## 4. Discussion

Although the clinical manifestations of each type of otitis media are different, surgery remains the treatment approach for both CSOM and middle ear cholesteatoma. There are slight differences in the use of antibiotics for treating the two types of otitis media, and the appropriate antimicrobial agent selection is solely based on ear secretion culture and drug sensitivity testing. In practical clinical work, the ear secretions' microbial culture results often do not meet the purpose of curing otitis media [17]. Clinicians rarely treat CSOM and middle ear cholesteatoma differently and do not select individualized treatments. Thus, there are limited studies on the detailed bacteriological differences between chronic otitis media and middle ear cholesteatoma.

In almost all molecular studies on the bacteriology of chronic otitis media, secretion swabs are collected from the middle ear cavity or the outer ear canal for gene sequencing. However, the collected secretions can be contaminated by bacteria in the external auditory canal or can be affected by the acquisition process. This may lead to false-positive results, and thus, these studies do not accurately reflect the true bacteriology of chronic otitis media [12, 18, 19]. Simultaneously, bacterial biofilm formation, like in many chronic inflammatory diseases, severely limits the ability to obtain positive results by conventional bacterial culture. Consequently, these analyses of chronic otitis media do not reflect the true clinical situation [20, 21].

The use of gene sequencing might be an alternative approach for analyzing unusual or dominant flora in diseased tissue. Consequently, this approach may be beneficial for the study of the pathogenesis of otitis media. In this prospective study, high-throughput gene sequencing of CSOM and cholesteatoma tissues was performed. Bacterial species abundance and diversity differed between the two types of otitis media. The bacterial species abundance and diversity of the cholesteatoma group were greater than those of the CSOM group. This finding is congruent with previous studies [13]. Collectively, data from these studies suggests that the condition of bacterial infection in the middle ear in cholesteatoma may be different and more complex than that of CSOM.

The current study revealed that the bacterial community composition in the middle ear lesion tissue of cholesteatoma was significantly more complex than that of CSOM. The cholesteatoma group lesions contained numerous Gram-positive and Gram-negative bacteria, which might be associated with the patient's long-term illness, with the bacteria forming a unique microenvironment, a coexistence relationship, and biofilm. In contrast, the situation of CSOM lesions is relatively simple, with bacterial communities at all taxonomic levels (phyla, classes, orders, families, genera, and species) dominated by Gram-negative bacteria. These results indirectly explain why broad-spectrum antibiotics are sometimes effective in CSOM but not in middle ear cholesteatoma patients.

The current study's findings differ from previous bacteriological studies that reported that chronic otitis media usually produced only one or two kinds of bacteria. This phenomenon is due to the difficulties in cultivating various bacteria using conventional bacteriological techniques, meaning such studies cannot reflect the full picture of infections in patients. However, using high-throughput gene sequencing, the pathogenic bacteria detection rate in middle ear cholesteatoma lesions was significantly higher than in CSOM lesions. This phenomenon indicates that cholesteatoma has a higher bacterial species complexity, and it is not an infectious disease caused by a single pathogenic bacterial species. Cholesteatoma may therefore constitute a bacterial microenvironment, whereby the combination of multiple conditional pathogens leads to the continuous onset of clinical symptoms of middle ear cholesteatoma, and a series of complications eventually emerge. This finding warrants further attention in future research to identify the role of bacterial microenvironment formation in the pathogenic mechanism of middle ear cholesteatoma and eventually provide a basis for the prevention and early treatment of middle ear cholesteatoma.

## Figures and Tables

**Figure 1:** Venn diagram of OTUs of CSOM and cholesteatoma lesions.

**Figure 2:** Pie charts showing phylum breakdown of bacterial communities obtained from CSOM (a) and cholesteatoma (b) pathological tissues.

**Figure 3:** Bubble diagram of class level differences in bacterial communities of CSOM and cholesteatoma pathological tissues.

**Figure 4:** Bar plot diagram showing bacterial composition at the order level in CSOM and cholesteatomas pathological tissues.

**Figure 5:** Pie charts showing composition of bacterial communities at the family level in CSOM (a) and cholesteatoma (b) lesions.

**Figure 6:** Pie charts showing genus-level composition of bacterial communities in CSOM (a) and cholesteatoma (b) lesions.

**Figure 7:** Bar plot showing species composition of bacterial communities of CSOM and cholesteatoma lesions.

## Data Availability

The data used to support the findings of this study are available from the corresponding author upon request.
